# MicroRNA-214 Suppresses Oncogenesis and Exerts Impact on Prognosis by Targeting PDRG1 in Bladder Cancer

**DOI:** 10.1371/journal.pone.0118086

**Published:** 2015-02-23

**Authors:** Jinfeng Wang, Xin Zhang, Lili Wang, Yongmei Yang, Zhaogang Dong, Haiyan Wang, Lutao Du, Chuanxin Wang

**Affiliations:** 1 Department of Clinical Laboratory, Qilu Hospital, Shandong University, Jinan, Shandong Province, China; 2 Department of Clinical Laboratory, Linyi People’s Hospital, Linyi, Shandong Province, China; Michigan State University, UNITED STATES

## Abstract

MicroRNA-214 (miR-214) has been reported to be dysregulated in human bladder cancer tissues. We aimed to investigate the clinical correlation, biological significance and molecular network of miR-214 in bladder cancer. Our results showed miR-214 was down-regulated in bladder cancer tissues and significantly associated with tumor stage, lymph node status, grade, multifocality, history of non-muscle-invasive bladder cancer (NMIBC). Moreover, miR-214 could serve as an independent factor of recurrence-free survival (RFS) and overall survival (OS) for patients with muscle-invasive bladder cancer (MIBC). Restoration of miR-214 expression in bladder cancer cell lines inhibited cell proliferation, migration, invasion and markedly promoted apoptosis. Dual-luciferase reporter assay recognized PDRG1 as direct downstream target gene of miR-214. PDRG1 was significantly increased in tumors low of miR-214 and knockdown of PDRG1 mimicked the effects of miR-214 overexpression. Our findings manifest that miR-214 could exert tumor-suppressive effects in bladder cancer by directly down-regulating oncogene PDRG1 and suggest an appealing novel indicator for prognostic and therapeutic intervention of bladder cancer.

## Introduction

Bladder cancer is the fourth most common cancer diagnosed in developed countries and accounts for the second leading cause of death among patients with genitourinary tract malignancies worldwide [1, 2]. Although approximately 75% of cases are grouped as NMIBC with a relatively high 5-year survival rate [3, 4], other 25% of patients with MIBC are subjected to subsequent metastatic disease after the first aggressive treatment [5]. Investigating new therapeutic modalities and identifying prognostic biomarkers for bladder cancer based on novel molecular networks have become research hotspots recently.

microRNAs (miRNAs) represent a class of small, endogenous, non-coding, 22-nucleotides RNA molecules that function as post-transcriptional regulator by partially pairing with the 3′-untranslated regions (UTR) of target mRNAs, leading to mRNA degradation or translational repression [6, 7]. It has been firmly established that miRNAs can regulate >60% of human protein-coding genes [8] and play crucial roles in various physiopathologic processes [9, 10]. miRNAs have been identified either as tumor suppressors or oncogenes [11]. In view of their disease- and tissue-specific expression profiles and amazing regulatory potential, miRNAs are being appraised as fascinating biomarkers for cancer diagnosis and prognosis [12]. Previous reports have demonstrated aberrant regulation of miRNAs in bladder cancer and several miRNAs (*e*.*g*., miR-9, miR-182, miR-200b, miR-145 and miR-129) show prognostic value [13–17]. Further studies are demanded to decode the underlying regulatory pathways by which miRNAs participate in the carcinogenesis of bladder cancer and to identify miRNAs functioning as novel therapeutic targets or as prognostic biomarkers for bladder cancer.

Some studies have reported that miR-214 was up-regulated and contributed to disease progression and distant metastases in malignant melanoma [18, 19], whereas others have indicated that miR-214 was down-regulated and had a tumor-suppressive effect in cervical cancer [20], breast cancer [21] and human hepatocellular carcinoma [22]. The above evidence points out that miR-214 may play pivotal and diverse roles in oncogenesis of various tumor types, yet potential mechanisms of miR-214 are still not completely unraveled. So far, there have been little published papers involving the functional analysis and molecular network of miR-214 in bladder cancer, though a few miRNA profiling studies showed that miR-214 was dysregulated in bladder cancer [23, 24].

In this study, we assessed expression level of miR-214 in human bladder cancer tissues, analyzed its feasible prognostic relevance and performed relevant functional experiments. We discovered that miR-214 could inhibit bladder cancer cell proliferation, migration, invasion and exert essential proapoptotic function. Furthermore, the oncogene PDRG1 was verified for the first time as a direct downstream target of miR-214 in bladder cancer. This report implicated a tumor suppressor role and regulatory mechanisms for miR-214 in bladder cancer.

## Materials and Methods

### Cell culture

The nonmalignant SV-40 immortalized bladder epithelial cell (SV-HUC-1) and two bladder cancer cell lines (T24 and 5637) were purchased from the Type Culture Collection of the Chinese Academy of Sciences (Shanghai, China) on May 22, 2014 having passed the test of DNA profiling (short tandem repeats, STR). The SV-HUC-1 cells were cultured in F12K medium (Sigma-Aldrich, St Louis, MO, USA) supplemented with 10% fetal bovine serum (FBS; TBD, Tianjin, china) and the two bladder cancer cell lines were cultured in modified RPMI 1640 medium (Hyclone, Logan, UT) supplemented with 10% FBS (TBD, Tianjin, china) at 37°C in a humidified incubator (5% CO2).

### Patients and tissue samples

This study was approved by the Medical Ethics Committee of Qilu Hospital of Shandong University and Linyi People’s Hospital. All patients signed written informed consent before their enrollment. A total of 106 operation patients with pathologically confirmed primary bladder transitional cell carcinoma were recruited between January 2004 and August 2009 from Qilu Hospital of Shandong University (n = 45) and Linyi People’s Hospital (n = 61). Among these patients, 31 patients underwent transurethral resection of bladder tumor and 75 patients underwent radical cystectomy. None of the patients had received preoperative therapy. Adjacent normal bladder tissues were obtained from regions outside the tumor margin (>5cm) in patients. All tissues were macro-dissected within 15 minutes after surgical resection, confirmed by pathological analysis of sequential frozen sections, and then stored at -80°C until use. The stage and grade of the tumors were evaluated in line with the Union for International Cancer Control 2009 TNM system [25] and 2004 WHO classification system [26] respectively. All patients were followed up by clinic visits every 3 months during the first 2 years, every 6 months for 2 years, and every year thereafter. RFS and OS were defined as the time interval between initial surgical resection and date of event or last follow-up.

### RNA isolation, cDNA synthesis and quantitative real-time PCR (qRT-PCR)

Total RNA was extracted from tissues or cells using TRIzol reagent (Invitrogen, Carlsbad, CA, USA) in accordance with the manufacturer’s protocol. The quantity and quality of RNA were checked with BioPhotometer plus (Eppendorf AG, Hamburger, Germany). For the detection of PDRG1, cDNA was synthesized by using a ReverTra Ace qPCR RT Kit (TOYOBO, Osaka, Japan). For miR-214, RNA was reverse transcribed using M-MLV reverse transcriptase (Invitrogen, Carlsbad, CA) and specific reverse transcription primer (RiboBio, Guangzhou, China). The expression levels of miR-214 and PDRG1 were quantified by way of qRT-PCR using Realtime PCR Master mix kit (TOYOBO, Osaka, Japan) and ABI 7500 real-time PCR system (Applied Biosystems, Foster city, USA) with snRNA U6 as their endogenous reference gene. The PCR reaction consisted of an initial denaturation step (95°C for 60s), 48 cycles (95°C for 15s, 60°C for 30s, 72°C for 45s) and melting curve analysis. The 2^-ΔΔCT^ method was performed to calculate the relative expression and expression levels of negative controls were used as calibrator.

### Mature miRNA or siRNA transfection

Bladder cancer cells were cultured at 3 × 10^4^ cells/well in 96-well plates or 1 × 10^5^ cells/well in 24-well plates or 5 × 10^5^ cells/well in 6-well plates in growth medium without antibiotics for approximately 24 hours until reaching 80% confluence and transiently transfected with miRNA mimics (Ribobio, Guangzhou, China) or siRNA (Ribobio, Guangzhou, China) using Lipofectamine 2000 (Invitrogen, Carlsbad, CA) according to the manufacturer’s instructions. miR-214 mimic and miR-negative control (miR-NC) mimic were used in the gain-of-function experiments, whereas si-PDRG1 and si-negative control (si-NC) were used in the loss-of-function experiments. To ensure actual transfection, qRT-PCR was carried out to detect transfection efficiencies in every experiment 24 hours later. For proliferation, wound-healing, migration, invasion and apoptosis assays, cells were harvested 24 hours after transfection. For western blot assay, cells were collected 48 hours posttransfection.

### Cell proliferation assay

According to the manufacturer’s protocol, the cell proliferation was detected at 24, 48, 72 and 96 hours after transfection by use of WST-8 staining with Cell Counting Kit-8 (Byotime, Haimen, China).

### Apoptosis assay

Bladder cancer cells were harvested, washed in cold PBS, resuspended, double stained with FITC-Annexin V/ propidium iodide Apoptosis Detection Kit (BestBio, Shanghai, China) according to the manufacturer’s recommendations and immediately analyzed by a flow cytometry (BD FACSCanto II, BD Biosciences, San Jose, USA).

### Wound-healing assay

Cells were plated in 6-well dishes with serum containing medium until subconfluence and serum-starved for 24 hours, then the cell monolayer was scratched across the center of the plates after the cells had reached confluence using a P-20 micropipette tip [27]. The initial gap length (0 hour) and the residual gap length at different time points (6, 12 and 24 hours) after wounding were photographed (200×) and calculated under IX71 inverted microscope (Olympus, Tokyo, Japan).

### *In Vitro* migration and invasion assays

Bladder cancer Cells in serum-free medium were placed into the upper chamber of the insert with 8-mm pores in 24-well tissue culture plates (Corning costar, NY, USA) with or without matrigel (BD Bioscience, Bedfold, MA, USA). Modified RPMI 1640 medium containing 10% FBS in the lower chamber served as the chemoattractant. After 24 hours of incubation, cells adhering to the lower membrane were washed, fixed and stained with 0.1% crystal violet and 20% methanol, imaged (400×), and counted using IX71 inverted microscope (Olympus, Tokyo, Japan).

### Dual-luciferase reporter assay

The pmiR-REPORT vectors (RiboBio, Guangzhou, China) were constructed with wild type (WT)-PDRG1 sequences or mutant (MUT)-PDRG1 sequences inserted between the hRluc and the hLuc gene. Bladder cancer cells in 96-well plates were co-transfected with miR-NC/miR-214 mimics and WT- PDRG1 3′-UTR vector/MUT- PDRG1 3′-UTR vector using Lipofectamine 2000 (Invitrogen). The activities of Renilla and firefly luciferases in cell lysates were measured using the Dual-Luciferase assay kit (Promega, Madison, WI) and the quotient of Renilla/firefly luciferase activities (Rluc/Luc) were considered as normalized data.

### Western blot

Lysis buffer (Beyotime, Haimen, China) was used to extract total protein from bladder cancer cells and concentration of protein was determined with Enhanced BCA Protein Assay Kit (Byotime, Haimen, China). Protein lysate was separated by SDS-PAGE and transferred onto PVDF membrane. After being blocked, the membranes were incubated with anti-PDRG1 rabbit mAb (1:1000; Abcam, Cambridge, MA, USA) or anti-β-actin mouse mAb (1:500; SantaCruz Biotechnology, Santa Cruz, CA) overnight at 4°C, then labeled with horse reddish peroxidase (HRP)-conjugated secondary antibodies (1:5000; Santa Cruz Biotechnology). Specific complexes were visualized with chemiluminescence HRP substrate (Millipore, Little Chalfont, UK).

### Target gene search for miR-214

To identify potential target genes of miR-214, we took advantage of an integrated bioinformatics analysis, starBase v 2.0 (http://starbase.sysu.edu.cn/targetSite.php), which can jointly use five public available algorithms (including targetScan, picTar, PITA, RNA22 and miRanda).

### Statistical analysis

All statistical analyses and graphing were performed using SPSS version 17.0, GraphPad Prism software and Microsoft excel. Significant differences between independent groups were calculated by Mann-Whitney U test, Kruskal-Wallis test or Student’s t-test. The Wilcoxon test was used to compare miR-214 expression in paired bladder cancer tissues and adjacent normal tissues. RFS and OS curves were determined by the Kaplan-Meier method and the survival differences of patients in sub-groups were evaluated by the log-rank test. Independent prognostic factors for survival prediction were estimated by Cox regression multivariate analysis. Spearman’s rank correlation analysis was applied to calculate the relationship between miR-214 and PDRG1. *P* < 0.05 was considered statistically significant.

## Results

### miR-214 is frequently attenuated in bladder cancer which is embroiled in cancer progression

We detected the expression level of miR-214 in 106 pairs of human bladder cancer frozen tissues and matched adjacent normal specimens by qRT-PCR and discovered that miR-214 was significantly underexpressed in bladder cancer tissues (*P* < 0.001) with the median expression level ten-fold lower than that of the noncancerous specimens (median expression = 0.084 and 0.864, respectively) (Fig. 1A). In addition, 74% of bladder cancer tissue samples showed more than two-fold lower miR-214 level compared to matched normal tissues (Fig. 1B and 1C). We further assessed the correlation between miR-214 expression in bladder cancer tissues and clinicopathologic features (Table 1) and observed that the attenuated miR-214 expression was significantly associated with higher tumor stage (*P* < 0.001), higher lymph node status (*P* < 0.001), higher grade (*P* < 0.001), multifocality (*P* = 0.003) and history of NMIBC (*P* = 0.033). Nevertheless, no significant correlation was found between miR-214 expression and other clinicopathological characteristics. These findings manifest that miR-214 may play a tumor-suppressive role in bladder cancer and its downregulation be embroiled in cancer progression.

**Fig 1:** miR-214 expression was frequently attenuated in bladder cancer tissues and associated with poor progonosis. **(A)** Expression level of miR-214 was determined by means of qRT-PCR and normalized against U6 RNA, an endogenous control, in 106 pairs of human bladder cancer tissues (BC) and matched adjacent normal tissues (NT). ***P < 0.001, Wilcoxon test, n = 106. (**B**) The attenuated expression of miR-214 was found in 74% (78 of 106) of bladder cancer tissues compared with adjacent normal specimens. (**C**) Relative expression of miR-214 was presented as log_2_ fold change (BC/NT) and the log_2_ fold change was defined as follows: <1, underexpression; >1, overexpression; the remaining was defined as unchanged. (**D**) Kaplan-Meier RFS and OS curves based on the miR-214 expression levels of patients with bladder cancer. The cut-off point was the median miR-214 expression level in the bladder cancer tissue samples. (**E**) Kaplan-Meier RFS and OS curves based on the miR-214 expression levels of patients with MIBC. The cut-off point was the median miR-214 expression level in the MIBC tissue samples.

**Table 1:** Clinicopathologic parameters and expression of miR-214 and PDRG1 in bladder cancer.

Variables	No. of cases	miR-214 expression [median (range)]	*P*	PDRG1 expression [median (range)]	*P*
Gender			0.368		0.012
Male	89	0.0841(0.0012–3.1123)		0.0053(0.0000–0.0261)	
Female	17	0.0419(0.0075–2.8011)		0.0146(0.0000–0.0262)	
Age			0.615		0.234
<57 years	50	0.0875(0.0012–3.1123)		0.0052(0.0000–0.0262)	
≥57 years	56	0.0576(0.0012–2.8011)		0.0066(0.0000–0.0261)	
Smoking status			0.238		0.084
non-smoker	55	0.1444(0.0012–3.1123)		0.0049(0.0000–0.0261)	
smoker	51	0.0499(0.0013–1.7630)		0.0075(0.0000–0.0262)	
History of NMIBC			0.033		0.128
No	14	0.0101(0.0012–0.6694)		0.0092(0.0003–0.0261)	
Yes	92	0.0978(0.0012–3.1123)		0.0062(0.0000–0.0262)	
Size			0.220		0.578
<3.6 cm	53	0.1443(0.0012–2.8011)		0.0064(0.0000–0.0216)	
≥3.6 cm	53	0.0524(0.0012–3.1123)		0.0063(0.0000–0.0262)	
Multifocality			0.003		0.111
No	70	0.1445(0.0012–3.1123)		0.0052(0.0000–0.0261)	
Yes	36	0.0185(0.0013–1.1559)		0.0089(0.0000–0.0262)	
Associated Cis			0.861		0.350
No	97	0.0841(0.0012–3.1123)		0.0063(0.0000–0.0262)	
Yes	9	0.0524(0.0013–1.6853)		0.0106(0.0021–0.0226)	
Grade			<0.001		0.001
Low	25	0.7637(0.0033–3.1123)		0.0035(0.0000–0.0189)	
High	81	0.0360(0.0012–1.1559)		0.0078(0.0000–0.0262)	
Tumor stage			<0.001		<0.001
Ta	12	0.7877(0.6395–3.1123)		0.0046(0.0000–0.0189)	
T1	19	0.4237(0.0033–2.2008)		0.0059(0.0000–0.0261)	
T2	25	0.1348(0.0012–1.1559)		0.0066(0.0000–0.0196)	
T3	25	0.0256(0.0023–0.9965)		0.0085(0.0000–0.0197)	
T4	25	0.0091(0.0029–0.0627)		0.0136(0.0000–0.0262)	
Lymph node status			<0.001		<0.001
N0	74	0.3373(0.0012–3.1123)		0.0044(0.0000–0.0261)	
N1	10	0.0124(0.0067–0.0419)		0.0198(0.0000–0.0216)	
N2	13	0.0122(0.0012–0.1145)		0.0127(0.0001–0.0262)	
N3	9	0.0042(0.0029–0.0419)		0.0109(0.0043–0.0243)	

### miR-214 serves as an independent prognostic predicator for patients with MIBC

During the follow-up, 54.7% (58 of 106) patients with bladder cancer experienced recurrence and the 5-year overall survival rate was 61.3% (65 of 106). The median follow-up of RFS and OS were 57.5 months (range, 0.5–79 months) and 62 months (range, 1–79 months) respectively. Kaplan-Meier survival curve revealed that bladder cancer patients with low miR-214 expression underwent significantly shorter RFS (log-rank test = 26.207; *P* < 0.0001) and OS (log-rank test = 45.174; *P* < 0.0001) than those with high expression (Fig. 1D), while multivariate Cox regression analysis showed that miR-214 was neither independent prognostic variable of RFS (*P* = 0.269) nor OS (*P* = 0.397) for bladder cancer patients.

Then, we performed separate analysis for the NMIBC and MIBC tumors. In the NMIBC group, after a median follow-up of 59 months (range, 42–79months), 54.8% of NMIBC patients (17/31) presented recurrence, but miR-214 neither predicted RFS nor OS when deregulated by Kaplan-Meier analysis. In the MIBC group, after a median follow-up of 32 months (range, 0.5–76 months), local or metastatic relapse was observed for 54.7% of the 75 MIBC patients (41/75), who all died. The 5-year overall survival rate was 45.3% (34 of 75) and the median follow-up of OS was 35 months (range, 1–76 months). Kaplan-Meier survival analysis revealed that decreased expression of miR-214 was significantly associated with poorer prognosis in terms of both RFS (log-rank test = 14.214; *P* = 0.0002) and OS (log-rank test = 13.797; *P* = 0.0002) (Fig. 1E). Furthermore, among the various clinicopathological parameters investigated in this study, age, history of NMIBC, tumor stage and lymph node status were significantly associated with outcome of MIBC at a significance level of 5% in univariate analysis. Multivariate Cox regression analysis including age, history of NMIBC, tumor stage, lymph node status and miRNA-214 showed that stage, lymph node status and miRNA-214 were independent prognostic predicators of RFS and OS for MIBC (Table 2).

**Table 2:** Factors affecting RFS and OS of MIBC patients in multivariate Cox proportional hazards regression analysis. sdddwwwwwwwwwwwwwwwwwwwwwwwwwwwwwwz

Prognostic factors	Recurrence-free survival			Overall survival		
	RR	95.0% CI	*P*	RR	95.0% CI	*P*
Age	1.549	0.755–3.176	0.232	1.483	0.733–3.000	0.273
Tumor stage	4.397	2.506–7.716	<0.001	3.880	2.245–6.706	<0.001
Lymph node status	2.934	2.049–4.200	<0.001	2.587	1.825–3.667	<0.001
History of NMIBC	1.149	0.483–2.734	0.753	1.046	0.447–2.449	0.918
miR-214	0.178	0.072–0.443	<0.001	0.230	0.097–0.547	<0.001

### miR-214 reintroduction suppresses oncogenicity *in vitro*

First, the expression level of mature miR-214 was found to be significantly down-regulated in bladder cancer cells compared with that in SV-HUC-1 by using qRT-PCR (Fig. 2A). To investigate the potential tumor suppressive role of miR-214, then we reintroduced miR-214 in bladder cancer cell lines followed by functional assays. Relative miR-214 expression in T24 and 5637 cells transfected with miR-214 mimic was 22319 and 10276 times higher than that transfected with miR-NC mimic confirmed by way of real-time PCR 24 hours posttransfection (Fig. 2B). As indicated in Fig. 2C, significant proliferation inhibitions were observed in miR-214-enhanced cells compared with control by Cell Counting Kit-8 assay. We also observed that apoptotic cell proportion was significantly increased upon miR-214 restoration compared with miR-NC by flow cytometry (Fig. 2D), indicating a proapoptotic role of miR-214 in regulating carcinogenesis. Moreover, bladder cancer cells overexpressing miR-214 displayed a significant reduction in migration ability in comparison with the controls by the wound healing assay (Fig. 3A) and transwell migration assay (Fig. 3B). As shown in Fig. 3C, transwell invasion assay with matrigel coating presented that miR-214 reexpression also significantly impaired the invasion ability of both cell lines. It is noteworthy that the incubation time for migration and invasion assays was within 24 hours after transfection, during which growth of bladder cancer cells was not affected by miR-214. So the inhibitory effects on cell migration and invasion were not caused by decrease in cell numbers. These observations demonstrate that miR-214 reintroduction suppresses the oncogenicity of bladder cancer cells *in vitro*.

**Fig 2:** miR-214 reintroduction inhibited cell proliferation and promoted apoptosis *in vitro*. (**A**) The miR-214 expression was significantly downregulated in bladder cancer cell lines than that in normal bladder cell line (SV-HUC-1). (**B**) Relative expression of miR-214 after miRNA mimic transfections as determined by qRT- PCR. (**C**) Cell viability assay in mock/miR-NC/miR-214 transfected bladder cancer cells (statistical analysis between miR-NC and miR-214: ***P < 0.001, t-test, n = 4). (**D**) Flow cytometry analysis showed that enforced expression of miR-214 significantly promoted apoptosis. Error bars correspond to mean ± standard error of the mean (SEM). ***P < 0.001, t-test, n = 6.

**Fig 3:** miR-214 restoration inhibited cell migration and invasion *in vitro*. (**A**) Wound healing assay, (**B**) Transwell migration assay and (**C**) Transwell invasion assay in mock/miR-NC/miR-214 transfected bladder cancer cells. Error bars correspond to mean ± SEM. ***P < 0.001, t-test, n = 6.

### Oncogene PDRG1 is a direct downstream target of miR-214

Since miRNA usually exerts its role by inhibiting the expression of downstream target genes, we further looked for the targets of miR-214 to elucidate the underlying mechanism of its antitumorigenic effects. Integrated bioinformatics analysis (targetScan, picTar, PITA and miRanda) demonstrates that PDRG1 contains one potential complimentary miR-214-binding site on its 3′-UTR (Fig. 4A). Given that, we first constructed pmiR-REPORT luciferase vectors containing wild-type or mutant 3^’^-UTR of PDRG1 inserted between the hRluc and the hLuc gene, and then carried out Dual-Luciferase reporter assay by cotransfecting above vectors with miR-214 mimics or miR-NC into bladder cancer cells. As shown in Fig. 4B, miR-214 significantly suppressed the relative luciferase activity of the reporter containing wild-type 3′-UTR but not the mutant reporter, signifying that PDRG1 is a direct downstream target for miR-214 in bladder cancer cells.

Consistent with this, depressed endogenous expression of PDRG1 in both mRNA and protein levels were observed in miR-214 reexpressed bladder cancer cells (Fig. 4C and 4D). Moreover, there was an inverse correlation between miR-214 and the PDRG1 expression in bladder cancer tissues (Fig. 4E). Taken together, our results forcefully verify that miR-214 negatively regulates PDRG1 expression by directly binding to its 3′-UTR complimentary sequences.

**Fig 4:** miR-214 negatively regulated PDRG1 expression by directly binding to its 3′-UTR complimentary sequences. (**A**) Sketch of the presumptive miR-214 binding sequences in PDRG1 3′-UTR and structure of wild-type or mutant PDRG1 pmiR-REPORT vectors. The mutant binding site was italicized and underlined. (**B**) Dual-Luciferase activity assay was performed in bladder cancer cells cotransfected with miR-NC/ miR-214 and pmiR-REPORT vectors containing WT- PDRG1 3′-UTR/ MUT-PDRG1 3′-UTR sequences. Data were displayed as normalized fold change in relative luciferase activity (Rluc/Luc). Error bars correspond to mean ± SEM. ***P < 0.001, t-test, n = 6. (**C**) The PDRG1 mRNA was down-regulated in bladder cancer cells transfected with miR-214 by qRT-PCR. Error bars correspond to mean ± SEM. ***P < 0.001, t-test, n = 6. (**D**) Western blot results of endogenous PDRG1 protein expression in bladder cancer cells transfected with miR-NC/ miR-214 with β-actin as a loading control. (**E**) Spearman’s correlation analysis indicated an inverse correlation between miR-214 expression and PDRG1 mRNA levels in bladder cancer tissues.

Compared to matched normal tissues, PDRG1 was significantly overexpressed in 81% of bladder cancer tissues detected by qRT-PCR (*P* < 0.001). In addition, we evaluated the correlation between PDRG1 expression in bladder cancer tissues and clinicopathologic parameters (Table 1) and discovered that the up-regulated PDRG1 expression was significantly associated with higher tumor stage, higher lymph node status, higher grade and gender. Kaplan-Meier survival curve showed that bladder cancer patients with high PDRG1 expression suffered significantly shorter RFS (log-rank test = 6.578; *P* = 0.010) and OS (log-rank test = 8.990; *P* = 0.003) than those with low expression, while multivariate Cox regression analysis demonstrated that PDRG1 was neither independent prognostic variable of RFS (*P* = 0.457) nor OS (*P* = 0.145) for bladder cancer patients. Performing separate Kaplan-Meier analyses for the NMIBC and MIBC tumors, PDRG1 neither predicted RFS nor OS when dysregulated in both groups.

### PDRG1 knockdown recapitulates the effects of miR-214 reexpression in bladder cancer cells

Aiming to investigate whether miR-214 exerts its antitumorigenic functions primarily through PDRG1, we treated bladder cancer cells with PDRG1 siRNA followed by functional assays. The knockdown effect was confirmed by RT-PCR and western blot analysis (Fig. 5A and 5B). Just as expected, significant proliferation inhibitions were observed in si-PDRG1 transfected cells compared with control (Fig. 5C). What’s more, apoptotic cell fractions were significantly increased upon PDRG1 knockdown in comparision with control as observed upon miR-214 reintroduction (Fig. 5D). The wound healing assay and transwell migration assay both indicated that si-PDRG1 significantly reduced the migration ability of bladder cancer cells (Fig. 6A and 6B). Noticeably, transwell assay with matrigel coating manifested that si- PDRG1 elicited an inhibitory effect on bladder cancer cell invasion compared with the control group (Fig. 6C). Above all, PDRG1 knockdown through siRNA technique mimicked the effects induced by enforced expression of miR-214, further indicating that PDRG1 may serve as a downstream functional mediator for miR-214.

**Fig 5:** PDRG1 knockdown inhibited cell proliferation and promoted apoptosis *in vitro*. (**A**) Relative expression of PDRG1 mRNA after siRNA transfections as determined by qRT- PCR. (**B**) Protein levels of PDRG1 were assessed by western blot in si-NC/si- PDRG1 bladder cancer cells with β-actin as a loading control. (**C**) Cellular proliferation assay in bladder cancer cells transfected with mock/si-NC/si-PDRG1 (statistical analysis between si-NC and si-PDRG1: ***P < 0.001, t-test, n = 4). (**D**) Flow cytometry analysis indicated that PDRG1 knockdown significantly promoted apoptosis. Error bars correspond to mean ± SEM. ***P < 0.001, t-test, n = 6.

**Fig 6:** PDRG1 knockdown inhibited cell migration and invasion *in vitro*. (**A**)Wound healing assay, (**B**) Transwell migration assay and (**C**) Transwell invasion assay in bladder cancer cells transfected with mock/si-NC/si-PDRG1. Error bars correspond to mean ± SEM. ***P < 0.001, t-test, n = 6.

## Discussion

In the current study, we verify for the first time a vital tumor suppressor, miR-214, that functions importantly in pathogenesis of bladder cancer. miR-214 was significantly down-regulated in tumorigenic bladder cancer cell lines compared with nonmalignant immortalized bladder epithelial cell line. Attenuation of miR-214 expression was assessed in approximately 74% of bladder cancer tissues and associated with higher tumor stage, higher lymph node status, higher grade, multifocality and history of NMIBC, suggesting that miR-214 may be embroiled in cancer progression. Our data are consistent with that of several studies as follows. For instance, miR-214 suppressed growth and invasiveness of cervical cancer cells by targeting UDP-N-acetyl-α-D-galactosamine [20]. Decreased miR-214 levels in breast cancer cells coincided with increased cell proliferation, invasion and accumulation of the Polycomb Ezh2 methyltransferase [21]. Downregulation of miR-214 contributed to tumor angiogenesis by inducing secretion of the hepatoma-derived growth factor in human hepatoma [22]. miR-214 regulated enhancer of zeste homolog 2 and inhibited migration and invasion in human esophageal squamous cell carcinoma [28]. miRNA expressing profiling studies showed that miR-214 was down-regulated in malignant bladder tissue samples and significantly differentially expressed between NMIBC and MIBC [23, 24]. Nevertheless, miR-214 serving as oncogene had been found up-regulated in other human cancers such as ovarian, stomach, pancreatic, cervical, lung, nasopharyngeal and oral mucosal cancers and malignant melanomas [18, 19, 29–32]. It is noticeable that functional disparities of miR-214 in different types of cancer may result from its diverse target genes or distinction among tissue types and cellular circumstances. It has been reported that miRNA can be silenced by structural genetic alterations (such as genomic deletion and inactivating mutations), promoter DNA methylation and loss of histone acetylation [33, 34]. In addition, at least one copy of the miR-214 alleles was found to be deleted in 24% of primary breast tumors [21]. In our study, attenuated miR-214 expression resulting from genomic loss or other mechanisms coupled with increased PDRG1 level may provide new prognostic biomarkers for the intervention of bladder cancer.

In the process of assessing the prognostic significance of miR-214, we discovered that bladder cancer patients with low miR-214 expression had a significantly higher recurrence and shorter overall survival after surgery and multivariate analysis identified miR-214 as an independent prognostic factor for RFS and OS in patients with MIBC. Our findings presented that miR-214 dysregulation could serve as a novel prognostic biomarker for MIBC, just as it can be prognosticator in human hepatoma [22]. In addition, urinary levels of cell-free miR-214 have been reported to be an independent prognostic parameter for NMIBC recurrence [35]. Although the use of a large body of bladder tumors with a wide variety of grade and stage in our study, independent validation studies are needed to evaluate the performance of miR-214 before considering its use as potential biomarkers. However, prognostic relevance of postoperative adjuvant therapy was not explored in this study although it was widely considered helpful for prognosis of bladder cancer. For one thing, there was no uniform therapeutic schedule in all cases according to the National Comprehensive Cancer Network (NCCN) Clinical Practice Guidelines in Oncology for bladder cancer; for another, some patients did not receive or failed to complete the adjuvant therapy because of economic pressures or unbearable side effects.

*In vitro* functional studies demonstrated that reexpression of miR-214 in bladder cancer cells induced phenotypes consistent with decreased cellular proliferation, migration and invasion concomitant with increased apoptosis, confirming the tumor-suppressive role of miR-214 in bladder cancer. Apoptosis serves as a well-orchestrated natural barrier to cancer pathogenesis and limiting or circumventing apoptosis is generally recognized as one of the major hallmarks of tumorigenesis [36]. Here we demonstrated that miR-214 restoration markedly induced apoptosis, verifying the important proapoptotic role of miR-214. Several miRNAs have also been reported to directly or indirectly regulate apoptosis in bladder cancer [13, 37]. Altogether, the suppressive effects on bladder cancer cell growth and metastasis combined with proapoptotic role of miR-214 might make for the poor prognosis of bladder cancer patients with low expression of miR-214.

Integrated bioinformatics analysis (targetScan, picTar, PITA and miRanda) recognizes PDRG1 as miR-214 target gene. However, the interaction between miR-214 and PDRG1 has not been reported. Dual-luciferase reporter assay revealed that PDRG1 had a miR-214 binding site in its 3′ UTR and PDRG1 was inversely related to miR-214 expression in bladder cancer clinical specimens. Restoration of miR-214 lowered PDRG1 expression in both mRNA and protein levels, suggesting that miR-214 reduce PDRG1 expression by degrading its mRNA. PDRG1 knockdown recapitulated the effects of miR-214 overexpression, further illustrating that the anti-tumor role of miR-214 may be mediated primarily via oncogene PDRG1. Additionally, our results showed that PDRG1 promoted bladder cancer cell proliferation and metastasis, while restrained apoptosis. To sum up, these findings suggest that miR-214 regulate PDRG1 to exert its tumor-suppressive effects.

Thus far, miR-214-mediated regulation of PDRG1 has not been reported before and is a discovery of particular importance as the rarely studied PDRG1 could involve in regulating cellular stress response, cancer development and progress [38]. PDRG1, namely p53 and DNA damage-regulated gene, resides at the long arm of chromosome 20 and encodes a protein of 133 amino acids presenting within a distinct subcellular compartment in the cytoplasm [39]. p53 could downregulate PDRG1 expression while genotoxic stress upregulate PDRG1 expression in a p53-independent manner [38]. It has been reported recently that PDRG1 expression was upregulated in multiple malignancies including cancers of the colon, rectum, ovary, lung, stomach, breast and uterus compared to their respective matched normal tissues and PDRG1 knockdown in human colon cancer cells resulted in marked slowdown of tumor cell growth [38], which is in line with our findings. Our study also indicated that up-regulated PDRG1 expression was significantly correlated with higher tumor stage, higher lymph node status and higher grade, suggesting it has the potential to be a novel valuable tumor biomarker that could play a role in bladder cancer development and/or progression.

A limitation to this study was that we were unable to carry out an *in vivo* study and further mouse xenograft model will be conducive to inspecting the therapeutic value of miR-214 in bladder cancer.

In conclusion, this is the first report elaborating that miR-214, whose attenuated expression in bladder cancer tissues is associated with worse prognosis, functions as a tumor suppressor by negatively regulating oncogene PDRG1 expression. These findings enrich our understanding of the crucial roles of dysregulated miRNAs in molecular pathogenesis of bladder cancer and provide novel insights into developing potential alluring targets for prognostic and therapeutic interventions in bladder cancer.

## Supporting Information

S1 Fig Original uncropped blots for Fig. 4D. (TIF)

S2 Fig Original uncropped blots for Fig. 5B. (TIF)
